# RTA408 alleviates retinal ganglion cells damage in mouse glaucoma by inhibiting excessive autophagy

This article has been retracted.

**DOI:** 10.1371/journal.pone.0313446

**Published:** 2024-11-11

**Authors:** Hongmei Qian, Wei Chen, Guomei Yuan, Man Luo, Li Zhang, Biao Wu, Hanshi Huang, Jiahao Xu, Qiong Wang, Mengyun Li

**Affiliations:** 1 Department of Ophthalmology, Shaoxing People’s Hospital, Shaoxing, Zhejiang, China; 2 Medical Research Center, Shaoxing People’s Hospital, Shaoxing, Zhejiang, China; Doheny Eye Institute, UNITED STATES OF AMERICA

## Abstract

**Background:**

Glaucoma, characterized by a high incidence and significant ocular harm, has been elucidated through various mechanisms. Excessive autophagy leading to the loss of retinal ganglion cells (RGCs) is suggested as one potential cause for visual impairment in glaucoma.

**Methods:**

A glaucoma model was established through anterior chamber injection of silicone oil in mice. RTA408 and the positive control tafluprost were administered for intervention. The efficacy was preliminarily assessed by intraocular pressure measurement. HE staining and fluorescent staining were used to assess RGC loss, while fluorescent staining and western blot were employed to evaluate the expression of Nrf2. The role of autophagy in the pathogenesis of glaucoma was investigated by artificially modulating autophagy levels.

**Results:**

In glaucomatous mice, RTA408 significantly reduces the apoptosis levels of RGCs and decreases RGC loss. Further investigations reveal a notable upregulation of autophagy levels in glaucomatous mice, with RGC loss being associated with autophagy. RTA408 promotes the expression of Nrf2 and downstream antioxidant molecules, enhancing the antioxidant system while downregulating mitochondrial autophagy levels. This reduces RGC apoptosis and loss, demonstrating a protective effect against glaucoma.

**Conclusion:**

Autophagy mediates the occurrence of glaucoma in mice, promoting RGC apoptosis. RTA408 alleviates RGCs damage by inhibiting excessive autophagy in the context of glaucoma.

## 1. Introduction

Glaucoma is a severe ocular disease often associated with elevated intraocular pressure, which can ultimately lead to blindness. Its hallmark features include the gradual loss of retinal ganglion cells (RGCs) and their axons. The pathogenesis of glaucoma involves disturbances in the production, circulation, and drainage of aqueous humor, resulting in increased intraocular pressure [1]. Tafluprost reduce intraocular pressure through several mechanisms, including increasing uveoscleral outflow, promoting aqueous humor outflow, and improving ocular blood flow. Moreover, research has indicated a significant connection between glaucoma and oxidative stress. Prolonged elevated intraocular pressure may induce oxidative stress in the optic nerve head, leading to an excessive generation of reactive oxygen species that can damage optic nerve cells, trigger inflammation and neurodegenerative changes, ultimately resulting in visual impairment [2]. Additionally, the vision loss associated with glaucoma is also linked to optic nerve damage caused by autophagy [3].

Autophagy is a physiological process of cellular self-degradation and clearance. Through this process, cells can break down and degrade damaged or aging organelles, proteins, and other cellular components, thereby maintaining the stability of the cellular environment [4]. Under normal circumstances, autophagy is a beneficial cellular process as it aids in the removal of impaired organelles and proteins [5]. However, excessive autophagy can lead to the loss of cellular functions, such as mitochondria, and excessive protein degradation, ultimately resulting in cell apoptosis. Particularly in RGCs, excessive autophagy induces mitochondrial dysfunction. Normal mitochondrial function is crucial for RGCs, as they require substantial energy to maintain nerve impulse conduction. Excessive autophagy leads to mitochondrial dysfunction and inadequate energy supply, thereby damaging RGCs [6].

RTA 408, also known as omaveloxolone, is a second-generation synthetic triterpenoid and Nfe2l2 (Nrf2) activator. It treats various diseases by activating the Nrf2 signaling pathway, exhibiting pharmacological effects such as anti-inflammatory, antioxidant, and antitumor properties, while also improving mitochondrial function [7,8]. Recent research indicates that RTA 408 inhibits osteoclastogenesis and ameliorates osteoporosis by impeding the STING-dependent NF-κB signaling pathway [9]. In fibroblasts from patients with Friedreich’s ataxia induced by oxidative stress, RTA 408 protects the normal mitochondrial membrane potential and prevents oxidative death [10]. It activates Nrf2 and promotes mitochondrial biogenesis to reverse neuropathic pain [11]. Furthermore, positive effects of RTA 408 on cardiovascular function have been observed in a mouse model of Friedreich’s ataxia, including recovery of ejection fraction, stroke volume, and cardiac output. It significantly ameliorated cardiac oxidative stress, inflammatory response, and cardiomyocyte apoptosis in septic cardiomyopathy mouse models by activating Nrf2 [12]. The aforementioned studies confirm the potent anti-inflammatory and antioxidant effects of RTA 408, yet there is a lack of related research on RTA 408 in the context of glaucoma.

Therefore, this study aims to investigate the therapeutic effects of RTA408 on mouse glaucoma and its regulatory mechanisms on autophagy by establishing a mouse model of glaucoma. The study compares RTA408 with the positive control drug tafluprost to assess its efficacy in ameliorating mouse glaucoma.

## 2. Materials and methods

### 2.1. Animals and treatment

All experiments were conducted following the "Guidelines for the Care and Use of Animals" and approved by the Institutional Review Board of Shaoxing People’s Hospital. Healthy 5-week-old male C57BL/6 mice were obtained from Shanghai SLAC Laboratory Animal Co., Ltd., and housed in a specific-pathogen-free animal facility. Mice were provided with ample water and food, maintained on a 12-hour light-dark cycle, and acclimatized for one week before randomization into four groups: Control, Chronic Ocular Hypertension (COH), COH+Tafluprost, and COH+RTA408. The Control group received no treatment. In the COH group, mice were anesthetized with inhaled isoflurane, and a puncture was made at the limbal region of both eyes under a microscope using an insulin needle. Subsequently, silicon oil was injected into the anterior chamber through a small hole parallel to the lens, blocking aqueous humor circulation and forming an oil bubble with a diameter of approximately 2mm (Fig 1A). Subsequently, intraocular pressure was measured every other day using a tonometer (icare, Finland), and sustained pressures above 20 mmHg indicated the successful establishment of the COH mouse model. In the COH+Tafluprost group, after successful COH model establishment, one drop of Tafluprost (Shentian Pharmaceutical Co., Ltd., China) was instilled into each eye daily. In the COH+RTA408 group, following COH model establishment, mice were orally gavaged with 10 mg/kg/day of RTA408 in a 0.6 mg/ml solution [13].

**Fig 1:** RTA408 significantly reduces RGCs loss in glaucoma. A. Schematic representation of silicone oil blocking aqueous humor circulation. B. Graph showing the changes in intraocular pressure among different groups of mice. C. Statistical analysis of GCC thickness among different groups of mice. D. HE staining of the peripheral, para-central, central, and entire retinas of mice in various groups. E. Quantification of RGCs in the peripheral, para-central, and central regions of the retinas among different groups of mice. IOP, intraocular pressure. RGCs, retinal ganglion cells. HE, Hematoxylin and eosin. GCC, ganglion cell complex. *P < 0.05.

To validate the involvement of autophagy and the regulatory mechanisms of RTA408 on autophagy, we employed 3-MA for autophagy inhibition and rapamycin for mTOR blockade in mice. The experimental groups included: Control, COH, COH+RTA408, COH+RTA408+3MA, and COH+RTA408+Rapamycin. The procedures for the Control, COH, and COH+RTA408 groups were consistent with those described earlier. In the COH+RTA408+3MA group, 3-MA (10 mg/kg/day) was intraperitoneally injected concurrently with RTA408 administration to inhibit autophagy [14]. For the COH+RTA408+Rapamycin group, rapamycin (2.0 mg/kg/day) was intraperitoneally injected simultaneously with RTA408 administration to block mTOR [15]. The entire treatment protocol lasted for 14 days, with eye pressure monitored every two days. On the 14th day, mice were euthanized with excess isoflurane, and the eyeballs were collected for further analysis.

### 2.2 Detection of Serum Redox marker

After anesthetizing the mice with isoflurane, enucleate the eyeball and collect blood from the orbital cavity. Following coagulation, serum was obtained. The levels of redox marker Superoxide dismutase (SOD), Malondialdehyde (MDA) and glutathione (GSH) were measured using commercial assay kits, following the manufacturer’s instructions (Nanjing Jiancheng Bioengineering Institute, Nanjing, China).

### 2.3 Hematoxylin and Eosin (HE) staining

Fresh eyeball tissues were embedded in embedding medium for frozen sections and cut into 5 μm-thick frozen sections. The sections were stained with the Hematoxylin-Eosin staining kit (Beyotime, Haimen, China) to examine myocardial and colonic morphology. Images of stained slides were captured using a Leica DM3000 microscope (Leica, Wetzlar, Germany), and RGCs were quantified using Image-ProPlus6 software (Media Cybernetics, Rockville, MD, USA).

### 2.4 Fluorescent staining of RGCs cells

After thawing at room temperature, frozen sections were blocked with 10% bovine serum albumin (BSA) blocking solution at 37°C for 30 minutes. Subsequently, the sections were incubated overnight at 4°C with RBPMS Polyclonal antibody (15187-1-AP, Proteintech, Rosemont, IL, USA), followed by a 1-hour incubation with Alexa Fluor 488-conjugated secondary antibody (Proteintech, Rosemont, IL, USA). Nuclear staining was performed using DAPI. Images were acquired using a confocal microscope (Leica Stellaris, Wezler, Germany).

### 2.5 Western blot

Total protein was extracted from retinal tissues using RIPA lysis buffer (Beyotime, Haimen, China) containing phosphatase inhibitor cocktail II (MedChemExpress, New Jersey, USA). Equal amounts of protein were separated by SDS-PAGE, transferred onto a PVDF membrane, and blocked with 5% skimmed milk for 1 hour. The membrane was then incubated overnight with specific antibodies, including Anti-BAX (ab32503, Abcam, Cambridge, England), anti-BCL2 (ab182858, Abcam, Cambridge, England), anti-cleaved-caspases 3 (ab214430, Abcam, Cambridge, England), anti-phospho-LC3B (ab63817, Abcam, Cambridge, England), anti-Nrf2 (#AF0639, Affinity, Jiangsu, China), anti-NQO1 (ab80588, Abcam, Cambridge, England), Anti-HO1(ab305290, Abcam, Cambridge, England), PINK1 (DF7742, Affinity, Jiangsu, China), Parkin (ab77924, Abcam, Cambridge, England), p62 (ab109012, Abcam, Cambridge, England), Atg5 (ab108327, Abcam, Cambridge, England), and anti-β-actin (#4970, CST, Danvers, MA, USA). After incubation with secondary antibodies, bands were visualized using enhanced chemiluminescence (Beyotime, Haimen, China). Band quantification was performed using Image-ProPlus6 software (Media Cybernetics, Rockville, MD, USA).

### 2.6 Immunofluorescence staining of Nrf2 in vivo

Immunofluorescence staining of Nrf2 in vivo was performed following deparaffinization with xylene and rehydration through a graded ethanol series. The sections were then blocked with a 10% bovine serum albumin (BSA) solution at 37°C for 30 minutes. Subsequently, the sections were incubated overnight at 4°C with the Nrf2 antibody (#AF0639, Affinity, Jiangsu, China), followed by a 1-hour incubation with Alexa Fluor 594-conjugated secondary antibody (Proteintech, Rosemont, IL, USA). Finally, nuclear staining was conducted using DAPI. Images were acquired using a confocal microscope (Leica Stellaris, Wezler, Germany).

### 2.7 Statistical analysis

All data were expressed as mean±SEM (standard error of the mean). Statistical analysis was performed using SPSS 22.0 software (SPSS Inc., Chicago, IL, USA), and graphs were generated using Prism 8 software (GraphPad, San Diego, USA). T-tests were used for statistical analysis between two groups. One-way or two-way ANOVA was used for comparisons among more than two groups, followed by Tukey’s post hoc analysis. A P-value less than 0.05 was considered statistically significant.

## 3.Result

### 3.1 RTA408 had no significant effect on intraocular pressure in the COH model

Through monitoring the intraocular pressure of mice, we evaluated the degree of relief provided by various intervention factors in mouse glaucoma. As shown in Fig 1B, the normal intraocular pressure of mice was maintained below 10 mmHg. However, following the obstruction of aqueous humor circulation by silicon oil, the intraocular pressure in the COH group mice remained above 25 mmHg, confirming the successful establishment of the chronic glaucoma model in mice. Treatment with Tafluprost significantly reduced intraocular pressure, as expected. However, the intervention with RTA408 did not effectively reduce intraocular pressure. This suggests that the therapeutic effect of RTA408 on glaucoma is not achieved by regulating intraocular pressure.

### 3.2 RTA408 reduced the loss of RGCs

Given that one characteristic of chronic glaucoma is the gradual loss of RGCs accompanied by a reduction in the thickness of the ganglion cell complex (GCC, includes the retinal nerve fiber layer (RNFL), the RGCs, and the inner plexiform layer) in the macular region, we observed the density of RGCs and the thickness of GCC in the retinas of mice in each group using HE staining and fluorescence staining. As shown in Fig 1C, the thickness of GCC in the COH group significantly decreased in the peripheral region, but both Tafluprost and RTA408 significantly reversed this phenomenon. Similarly, compared to normal mice, the density of RGCs significantly decreased in the peripheral region of the retina in the COH group, but the application of Tafluprost and RTA408 prevented the loss of RGCs. Similar observations were made in the para-central region of the retina. However, surprisingly, in the central region of the retina, although a reduction in RGCs was observed in the COH group, the application of Tafluprost and RTA408 did not significantly reverse the loss of RGCs (Fig 1D and 1E).

After performing immunofluorescence staining for RGCs, we observed similar phenomena. In the peripheral and para-central regions, sustained high intraocular pressure resulted in a significant reduction of RGCs, while both Tafluprost and RTA408 prevented the loss of RGCs. However, this effect was not significant in the central region (Fig 2A and 2B).

**Fig 2:** RTA408 significantly reduces RGCs loss. A. Immunofluorescence imaging of RGCs in the peripheral, para-central, central, and entire retinas of mice in different groups. B. Quantification of RGCs in the peripheral, para-central, and central regions of the retinas among different groups of mice. C-D. Western blot analysis showing the expression levels of BAX, BCL-2, and Cleaved Caspase-3. RGCs, retinal ganglion cells. *P < 0.05.

### 3.3 RTA408 reduced the level of apoptosis in RGCs

To further elucidate the reasons for the reduction in RGCs, we conducted an assessment of apoptosis levels in retinal tissue. The COH group exhibited a significant increase in Bax/BCL-2 ratio, along with a marked elevation in the expression of cleaved-caspases 3, strongly indicating an elevated level of RGCs apoptosis. Encouragingly, the use of Tafluprost and RTA408 both significantly reduced the apoptosis levels (Fig 2C and 2D).

### 3.4 RTA408 promotes the expression of Nrf2 and downstream antioxidant molecules

To further elucidate the mechanism by which RTA408 protects RGCs, we first used immunofluorescence to examine the expression of Nrf2 in retinal tissue. The results showed that Nrf2 expression was significantly increased after RTA408 intervention (Fig 3A). Next, we used western blotting to detect the activation of the Nrf2-NQO1/HO1 pathway. In the COH group, due to disease-induced stress, Nrf2 expression had already begun to increase, but the downstream antioxidant molecules NQO1 and HO1 were depleted and reduced. Interestingly, after RTA408 intervention, Nrf2 expression was significantly upregulated, and downstream NQO1 and HO1 were also abundantly expressed (Fig 3B). We also examined key components of the body’s antioxidant system, including SOD and GSH, as well as the oxidative stress marker MDA, and found that RTA408 intervention significantly upregulated the levels of SOD and GSH while significantly reducing MDA content (Fig 3C). These results indicate that RTA408 activates Nrf2, enhances the body’s antioxidant system, and reduces oxidative stress levels.

**Fig 3:** RTA408 promotes Nrf2 expression. **A**. Immunofluorescence staining of Nrf2 in retinal tissues of mice from different groups. **B.** Western blot analysis of Nrf2 and downstream signaling pathway proteins in retinal tissues of mice from different groups. **C.** ELISA detection of serum SOD, MDA, and GSH levels in mice. *P < 0.05.

### 3.5 Autophagy is involved in the loss of RGCs in COH, and RTA408 rescues this phenomenon by modulating autophagic imbalance

To further explore the mechanisms underlying the reduction of RGCs and considering the crucial role of autophagy in neuronal cell damage, we assessed the involvement of autophagy in the development of COH. Compared to the control group, a significant upregulation of autophagy was observed in the COH group, strongly indicating the potential involvement of autophagy in the loss of RGCs (Fig 4A and 4B). To confirm the role of autophagy in this process, first we separately employed rapamycin and 3-methyladenine (3-MA) to enhance and inhibit autophagy, respectively. As expected, rapamycin intervention significantly upregulated autophagy levels, while 3-MA inhibited autophagy levels (Fig 4A and 4B). The robust increase in autophagy induced by rapamycin resulted in a significant reduction in the number of RGCs under elevated intraocular pressure. Conversely, when autophagy was strongly suppressed by 3-MA, RGCs were well-preserved under high intraocular pressure (Fig 5A and 5B), and immunofluorescence results confirmed this observation (Fig 6A and 6B).

**Fig 4:** Autophagy significantly increases RGCs loss. A. HE staining of the peripheral, para-central, central, and entire retinas of mice in different groups. B. Quantification of RGCs in the peripheral, para-central, and central regions of the retinas among different groups of mice. HE, Hematoxylin and eosin. RGCs, retinal ganglion cells. *P < 0.05.

**Fig 5:** Autophagy significantly increases RGCs loss. A. Immunofluorescence imaging of RGCs in the peripheral, para-central, central, and entire retinas of mice in different groups. B. Quantification of RGCs in the peripheral, para-central, and central regions of the retinas among different groups of mice. RGCs, retinal ganglion cells. *P < 0.05.

**Fig 6:** Autophagy significantly influences the apoptotic levels of RGCs in glaucomatous mouse eyes. **A-B.** Detection of the expression levels of BAX, BCL-2, and Cleaved Caspase-3 through Western blot analysis. RGCs, retinal ganglion cells. *P < 0.05.

Furthermore, our findings revealed that intervention with RTA408 significantly reduced apoptosis levels, and the upregulation of autophagy led to an increase in RGC apoptosis. Downregulating autophagy levels with 3-MA significantly alleviated RGC apoptosis. These results strongly suggest that autophagy hyperactivation may be a core factor contributing to the loss of RGCs (Fig 7A and 7B). Following RTA408 intervention, a significant downregulation of autophagy levels, as indicated by the detection of autophagic protein LC3, implies that RTA408 alleviates COH, at least in part, through the autophagic pathway (Fig 7A and 7B). In conclusion, autophagy participates in the loss of RGCs during the development of COH, and RTA408 can modulate autophagy levels, thereby reducing RGC apoptosis.

**Fig 7:** RTA408 inhibits excessive autophagy in the eyes of glaucomatous mice. A-B. Assessment of the expression levels of p-mTOR and LC3 through Western blot analysis. *P < 0.05.

### 3.6 RTA408 attenuates the mitophagy pathway

To further elucidate the specific autophagy pathway regulated by RTA408, we examined the proteins involved in the PINK1/Parkin-mediated mitophagy pathway. Surprisingly, in the COH group, mitophagy was significantly activated, but after RTA408 intervention, the levels of PINK1 and Parkin were downregulated, indicating that the mitophagy pathway was inhibited (Fig 8A).

**Fig 8:** RTA408 inhibits the mitophagy pathway. **A.** Western blot analysis of mitophagy-related molecules in retinal tissues of mice from different groups. *P < 0.05.

## 4.Discussion

In this study, we found that RTA408, while not significantly reducing elevated IOP in chronic ocular hypertension, significantly reduced the loss of RGCs. The protective effect of RTA408 on RGCs appears to be mediated through the reduction of RGC apoptosis. Further investigation revealed that autophagy was involved in the loss of RGCs during the COH process, and RTA408 improved RGC damage by inhibiting the excessive autophagy.

The main characteristic of glaucoma is elevated intraocular pressure, which may lead to the traction and deformation of the retinal nerve fiber layer, causing damage to RGCs. Elevated intraocular pressure can also restrict blood supply to the optic nerve, resulting in ischemia and hypoxia. This ischemic and hypoxic condition may lead to metabolic abnormalities in RGCs, increasing the sensitivity of cells to oxidative stress. Excessive production of reactive oxygen species may damage the cell membrane, proteins, and nucleic acids of RGCs, promoting the apoptosis process.Some studies suggest that inflammation is present in ocular tissues of glaucoma patients. Infiltration of inflammatory cells and release of inflammatory mediators may directly or indirectly affect RGCs, contributing to apoptosis. RTA408, as a potent anti-inflammatory and antioxidant molecule, has demonstrated protective capabilities in various diseases such as renal ischemia-reperfusion [16], asthma [17], neurological damage [18], and osteoporosis [4]. In our study, we found that RTA408 did not reduce intraocular pressure in chronic ocular hypertension, suggesting that the mechanism by which RTA408 protects RGCs might be independent of IOP reduction. We observed that although elevated IOP significantly increased the level of RGC apoptosis, treatment with RTA408 significantly alleviated RGC apoptosis and greatly preserved the number of RGCs. This has an important role in delaying vision loss.

Autophagy is a physiological process wherein cells undergo self-degradation and clearance. Through this process, cells can break down and degrade damaged or aging organelles, proteins, and other cellular components to maintain internal environmental stability [19]. This process is crucial for cell survival, development, and adaptation to environmental changes [20]. Autophagy is also believed to play a role in the pathogenesis of various diseases, including neurological disorders, cancer, and infectious diseases. In some cases, autophagy may be excessively activated, leading to abnormal cell death, while in other instances, insufficient autophagy may result in the accumulation of cellular waste. Therefore, maintaining autophagy at an appropriate level is particularly important [21,22]. More importantly, there is a close relationship between autophagy and oxidative stress. Oxidative stress can induce the activation of autophagy, which allows cells to increase autophagy to remove damaged mitochondria, oxidatively damaged proteins, and aggregates when subjected to oxidative damage, thereby reducing the generation of ROS and mitigating the effects of oxidative stress [23,24], However, excessive autophagy can sometimes occur, leading to damage to normal cells as well. Therefore, reducing the level of oxidative stress is also effective in decreasing the level of autophagy. In our study, hyperactive autophagy was observed in COH. Through artificially modulating autophagy levels, we further demonstrated that autophagy imbalance is a significant factor contributing to the loss of RGCs. Additionally, we found that heightened autophagy increases the level of RGC apoptosis, which may be a core reason for the reduction in RGC quantity. Rapamycin is a commonly used autophagy inducer that can further enhance already excessive autophagic activity, this may lead to the excessive degradation of cellular components, including important organelles and proteins, thereby impairing cell function. After intervention with RTA408, the expression of Nrf2 and downstream antioxidant molecules NQO1 and HO1 was significantly increased, enhancing the antioxidant system, while the level of autophagy was markedly inhibited, which is crucial for the preservation of RGCs.

The limitations and strengths of this study are worth exploring. Firstly, there are inherent differences between mouse disease models and human conditions, and responses to drugs may also vary. Therefore, these research findings need further support through additional relevant clinical trials. However, it is noteworthy that using mice in research allows better control of genetic backgrounds, uniform SPF-level living environments, circadian rhythms, and drug intervention compliance. These factors significantly impact the severity of glaucoma and autophagy levels. Thus, utilizing mice in the study substantially reduces errors caused by individual differences in lifestyle rhythms and genetic backgrounds. Secondly, as mentioned earlier, autophagy has a dual nature. While excessive autophagy is detrimental, the body requires autophagic responses to clear aging organelles. Therefore, controlling autophagy at an appropriate level is crucial. Although this study confirmed that RTA408 inhibits excessive autophagy, whether it affects the normal autophagic response in other organs was not explored in this study. Currently, there is a lack of relevant research reports on this matter, making it an important focus for future investigations. Thirdly, in this study, we also found that RTA408 had a better protective effect on RGCs in the peripheral and para-central regions of the retina, with no significant impact on the number of central RGCs. We believe that, on one hand, the greatest mechanical damage caused by lamina cribrosa movement occurs in the axons located in the peripheral part of the optic nerve, initiating RGC damage in the peripheral region, while the levels of oxidative stress and autophagy in the central cells may not be severe, resulting in less significant effects of RTA408. Secondly, the central RGCs are densely distributed with a large cell population, so even if RTA408 rescued some cells, the change in the overall number would be negligible. However, this is our hypothesis based on clinical experience, and the exact mechanisms require further investigation.

## Supporting information

S1 File The original uncropped and unadjusted images underlying all blot or gel results. https://figshare.com/s/690f05fd7f6e0e743a95.
(PDF)

S2 File The original plotting data. (XLSX)

## Abbreviations

RGCs: retinal ganglion cells
Nrf2: Nfe2l2
COH: chronic Ocular Hypertension
HE: Hematoxylin and Eosin
BSA: bovine serum albumin
GCC: ganglion cell complex
3-MA: 3-methyladenine
MDA: Malondialdehyde
SOD: Superoxide dismutase
GSH: Glutathione
